The article "Upregulated NLGN1 predicts poor survival in colorectal cancer" was published in 2021. Journal: BMC Cancer.

# Upregulated NLGN1 predicts poor survival in colorectal cancer

**DOI:** 10.1186/s12885-021-08621-x

**Published:** 2021-08-02

**Authors:** Qian Yu, Xiaojie Wang, Yinghong Yang, Pan Chi, Jianping Huang, Shengliang Qiu, Xin Zheng, Xiaowen Chen

**Affiliations:** 1 Department of Pathology, Union Hospital, Fujian Medical University, 29 Xin-Quan Road, Fuzhou, Fujian 350001 People’s Republic of China; 2 Department of Colorectal Surgery, Union Hospital, Fujian Medical University, 29 Xin-Quan Road, Fuzhou, Fujian 350001 People’s Republic of China

**Keywords:** Colorectal cancer, NLGN1, Survival

## Abstract

**Background:**

Neuroligin1 (NLGN1) is a main component of excitatory glutamatergic synapses complex and is important for synapse assembly and function. The clinical value of NLGN1 in colorectal cancer (CRC) is not clear.

**Methods:**

We obtained the expression data of 1143 CRC patients from 3 independent Gene Expression Omnibus (GEO) datasets (GSE32323, GSE24551, GSE39582) and The Cancer Genome Atlas (TCGA) to make the comparison of the NLGN1 expression level between CRC tissues and matched noncancerous tissues, and to evaluate its value in predicting survival of CRC patients. At the protein level, these results were further confirmed by immunohistochemical staining of 52 CRC samples in our own centre. Finally, the function of NLGN1 was explored by gene set enrichment analysis (GSEA).

**Results:**

Increased mRNA and protein levels of NLGN1 expression were associated with worse overall survival or recurrence-free survival in CRC patients from 2 GEO datasets, the TCGA database, and our cohort. In addition, multivariate regression analysis showed that NLGN1 was an independent poor prognostic factor of survival in patients with CRC in TCGA database (OR = 2.524, *P* = 0.010). Functional analysis revealed that NLGN1 was correlated with function involving the Hedgehog signaling pathway, mismatch repair process, and some material metabolism processes.

**Conclusions:**

This study is the first to implicate and verify NLGN1 as a new poor prognostic marker for CRC.

## Background

Colorectal cancer (CRC) has seen a obvious increase in the annual global incidence rate and is the third most common cancer worldwide [1]. Despite overall therapeutic improvements, CRC remains the fourth most common cause of cancer-related death [2]. A classic prognostic tool such as the tumor-node-metastasis (TNM) system is directly correlated with CRC patient’s survival or relapse [3] and is used for the determination of therapeutic strategies [4]. However, the prognosis varies greatly in patients within the same stage [5]. Besides, multiple options were recommended for patients with the same stage due to different prognosis. For instance, the National Comprehensive Cancer Network (NCCN) guidelines suggest different options, ranging from sole observation to several different adjuvant therapeutic regimens, for stage II patients after surgery of primary colon cancer [6]. Hence, molecularly based prognostic markers are needed to further distinguish risk levels within CRCs.

Neuroligin 1 (NLGN1) encodes a trans-synaptic protein that acts as a postsynaptic adhesion molecule involved in the regulation of glutamatergic transmission [7]. At excitatory synapses, NLGN1 mediates transsynaptic binding with neurexin [8] and was known to play a pivotal role in memory formation and modulation of memory strength [9]. Currently, diseases associated with NLGN1 in previous studies include autism [10], post-traumatic stress disorder [11] and schizophrenia [12]. The role of NLGN1 in cancer is largely unknown. Moreover, the expression level of NLGN1 in CRC tissues and its clinical value have never been studied. Therefore, the aim of this study was to determine NLGN1 expression in CRC tissues and to evaluate its prognostic value.

## Methods

### Analysis of bioinformatics databases

A total of 3 independent microarray datasets were obtained from the Gene Expression Omnibus (GEO) database (https://www.ncbi.nlm.nih.gov/geo/). The dataset GSE32323 [13] included mRNA genome arrays of 17 pairs of cancer and matched normal tissues from CRC patients. The dataset GSE39582 [14] included 443 CRC mRNA expression profiles from a high volume center. The dataset GSE24551 [15] included exon level expression profiles of 160 CRC tissues.

RNA sequencing (RNA-Seq) data from 465 patients with colon cancer were retrieved from the TCGA database. Cases without survival data or NLGN expression data were excluded (*n* = 27), leaving 438 patients included for further analysis. In addition, the Cbioportal (www.cbioportal.org) was used to extract the methylation data, copy number data, and mutation status data of NLGN1 from public datasets.

### Cohort in our Centre

To confirm the differential expression of NLGN1 in protein level between CRC and normal samples, immunohistochemistry (IHC) staining was performed on 52 colorectal cancer tissues and paired noncancerous tissues in our centre. All patients with pathology confirmed adenocarcinoma had received radical surgery between February 2012 and December 2013. Reception of neoadjuvant therapy was an exclusion criterion. Clinicopathological data of all patients was retrospectively collected. TNM stages were evaluated according to AJCC 7th [16].

### IHC staining

Formalin-fixed tissue specimens were embedded in paraffin. The NLGN1 protein expression in 52 CRC and paired adjacent normals were evaluated using IHC analysis. Anti-NLGN1 monoclonal antibody (NBP1–87888, NOVUS, USA) was used at a working concentration of 1:50. The scores were measured basing intensity and staining density. The results were condensed into four categories: negative (−), weakly positive (+), positive (++), and strongly positive (+++). High expression of NLGN1 was defined as a total score of ≥2 + .

### Gene set enrichment analysis (GSEA)

GSEA was performed to identify the function of NLGN1 using c2.cp.kegg.v5.2.symbols.gmt as the reference. Three datasets, including GSE24551, GSE39582, and TCGA were used. Patients with the top 50% and with the bottom 50% of the expression of NLGN1 were compared. |enrichment score (ES) | < 0.3 was deemed not significant. Gene size ≥15 were set as the cutoff criteria. The overlapping enriched hallmark signatures among these 3 databases were chosen.

### Statistical analysis

Categorical variables were compared using the chi-squared tests. Continuous variables were compared using Student’s t-test and paired t-tests, as appropriate. The cutoff value for NLGN1 expression was determined by X-tile 3.6.1 software (Yale University, New Haven, CT) [17]. Percent survival was calculated using the Kaplan-Meier method compared by log-rank test. Univariate Cox regression analysis was applied to estimate the Odd ratio (OR) for survival. Variables with *P* < 0.10 in univariate analysis were entered into multivariate analysis to confirm the independent prognostic factors. Significance was defined as *P* value of < 0.05. All statistical analyses were performed using SPSS software (ver. 17, SPSS Inc., Chicago, IL), GraphPad Prism Software (v7.0, Graphpad Software, La Jolla, CA) and R (ver. 3.5.1).

The recurrence-free survival (RFS) was defined as the time interval from surgical resection to the first recurrence or censored at 5 years. Disease-free survival (DFS) was defined as the time from surgical resection until the first documented progression of disease, death, or date of the last follow-up. Overall survival (OS) was defined as the time from surgery to either death or last follow-up.

Workflow of this study is shown in Fig. 1.

**Fig. 1:** The workflow of this study

## Results

### NLGN1 expression is upregulated in CRC

To determine the NLGN1 mRNA levels in CRC samples, we compared the NLGN1 mRNA expression between 17 CRC tissues and matched normals in GSE32323 dataset. The analysis revealed that NLGN1 expression was significantly increased in CRC tissues compared with that in matched mucosa (8.3 ± 0.3 vs. 8.1 ± 0.2, *P* = 0.032, Fig. 2A). IHC analysis was then performed to assess the NLGN1 protein levels in 52 pairs of CRC tissues and adjacent normals. The NLGN1 protein was expressed at higher levels in CRC tissues (total score: 2.2 ± 1.1) than in matched normals (total score: 1.6 ± 0.7; *P* < 0.0001, Fig. 2B). NLGN1 was mainly located in the cytoplasmic membrane of normal glandular cells and adenocarcinoma cells. Interestingly, ganglion cells had positive NLGN1 protein expression. Moreover, our IHC analysis revealed that the patients with perineural invasion had significantly higher NLGN1 expression than those without perineural invasion (7.6 ± 3.2 vs. 5.8 ± 3.8, *P* = 0.010, Fig. 2C). Due to limited sample size in our own patients, the trend toward a higher rate of high NLGN1 expression with perineural invasion was not significant (rate of high NLGN1 expression in perineural invasion vs. No perineural invasion: 75.0% vs. 39.6%, *P* = 0.395). The status of perineural invasion in CRC patients was provided in only the TCGA database among the 4 publicly available datasets. Of the 176 CRC patients with known perineural invasion status, the mRNA expression of NLGN1 in patients with perineural invasion was higher than that in patients without perineural invasion (5.4 ± 2.0 vs. 1.9 ± 0.4, *P* = 0.011). Illustrations of different NLGN1 expression levels in CRC tissues and normals are displayed in Fig. 3. In addition, a representative example of CRC cells with positive NLGN1 protein expression invading nerve bundles in the perineural space is shown in Fig. 4.

**Fig. 2:** The relationship between NLGN1 expression and clinical characteristics of CRC patients. NLGN1 mRNA was upregulated in CRC tissues compared with that in adjacent normals in (**A**) GSE32323 dataset and at the protein level in (**B**) our cohort. **C** The patients with perineural invasion had significantly higher NLGN1 expression than those without perineural invasion. **D** NLGN1 expression level was significantly higher in microsatellite stable (MSS) patients compared with that in microsatellite instable (MSI) patients

**Fig. 3:** Representative images of NLGN1 immunohistochemical analysis in CRC patients in our centre (magnification × 200). **A**-**B** Negative-weakly NLGN1 expression in CRC tissue; **C** Illustrations of NLGN1 protein expression in sections of non-cancerous mucosa (five-pointed star) adjacent to tumors (triangle); **D**-**E** Positive-strongly positive NLGN1 expression in CRC tissue; **F** Illustrations of NLGN1 protein expression in ganglion cells (arrowhead)

**Fig. 4:** Illustrations of CRC cells (star) with positive NLGN1 protein expression invading nerve bundles in the perineural space (triangle) (magnification × 200). **A** Hematoxylin-eosin staining; **B** Immunohistochemical staining

### Survival analysis based on NLGN1 expression

The value of NLGN1 in predicting survival of CRC patients was evaluated first in the GEO and TCGA at the RNA level. Table 1 showed the characteristics of patients in each included cohort. Each cohort was divided into two groups according to the cutoff point determined by X-tile. CRC patients with high NLGN1 expressions in GSE24551 had significantly decreased 5-year overall survival rates (5Y-OS) than those with low NLGN1 expression (45.2% vs. 74.8%, *P* = 0.0002, Fig. 5A). In GSE39582, high NLGN1 expressions were also associated with lower 5Y-OS and 5-year recurrence-free survival rates (61.2% vs. 72.4%, *P* = 0.037, Fig. 5B; 58.1% vs. 72.3%, *P* = 0.00006, Fig. 5D). The results were then confirmed in patients from TCGA (5Y-OS of high expression vs. low expression: 64.0% vs. 79.3%, *P* = 0.0009, Fig. 5C). At the protein level, IHC analysis was performed in patients from our centre. Survival analysis showed that CRC patients with high NLGN1 protein expression had worse 5-year disease-free survival than those with low NLGN1 protein expression (high expression vs. low high expression: 44.4% vs. 66.7%, *P* = 0.030, Fig. 5E).

**Table 1:** Clinical characteristics of patients in included databases and our cohort

Cohorts	Characteristics		Values	
GSE32323 dataset	TNM stage	I	2	(11.8)
		II	7	(41.2)
		III	5	(29.4)
		IV	3	(17.6)
GSE24551 dataset	TNM stage	II	90	(56.3)
		III	70	(43.8)
GSE39582 dataset	Gender	Male	288	(54.5)
		Female	240	(45.5)
	Age (years)		66.6 ± 13.4	
	TNM stage	0	4	(0.8)
		I	32	(6.1)
		II	246	(46.6)
		III	188	(35.6)
		IV	58	(11.0)
TCGA database	Gender	Male	234	(53.4)
		Female	204	(46.6)
	Age (years)		66.6 ± 13.0	
	TNM stage	I	73	(16.7)
		II	194	(44.3)
		III	99	(22.6)
		IV	61	(13.9)
		Missing	11	(2.5)
	Histological type	Adenocarcinoma	373	(85.2)
		Mucinous adenocarcinoma	60	(13.7)
		Missing	5	(1.1)
	Perineural invasion	No	131	(29.9)
		Yes	45	(10.3)
		Missing	262	(59.8)
	Tumor deposits	No	184	(42.0)
		Yes	38	(8.7)
		Missing	216	(49.3)
Our cohorts	Gender	Male	28	(53.8)
		Female	24	(46.2)
	Age (years)		65.4 ± 12.4	
	TNM stage	I	9	(17.3)
		II	14	(26.9)
		III	21	(40.4)
		IV	8	(15.4)
	Tumor location	Left colon	5	(9.6)
		Right colon	20	(38.5)
		Rectum	27	(51.9)
	Perineural invasion	No	48	(92.3)
		Yes	4	(7.7)
	Venus invasion	No	48	(92.3)
		Yes	4	(7.7)
	Tumor deposit	No	46	(88.5)
		Yes	6	(11.5)
	Tumor location	Left colon	5	(9.6)
		Right colon	20	(38.5)
		Rectum	27	(51.9)

**Fig. 5:** Increased NLGN1 expression predicted worse overall survival in CRC patients from **A** GSE24551, **B** GSE39582, and **C** TCGA. Higher NLGN1 levels were associated with significantly decreased recurrence-free survival rates in **D** GSE39582 and disease-free survival rates in **E** patients in our centre

### Multivariate analysis

Univariate analysis and multivariate analysis were performed. In RNA-seq data, NLGN1 was confirmed as an independent prognostic marker of poor OS in multivariate Cox regression analysis in the TCGA database (OR = 2.524, *P* = 0.010, Table 2). At the protein level, univariate analysis based on our cohort also revealed that NLGN1 was a poor prognostic indicator of DFS (OR = 2.368, *P* = 0.034, Table 3). Due to the small sample size, multivariate Cox regression analysis was not performed.

**Table 2:** Univariate and multivariate analyses of the prognostic factors of OS in CRC patients from TCGA database

Factors		Univariate analysis				Multivariate analysis			
		Odd ratio	95% CI		P value	Odd ratio	95% CI		P value
Age	(per year)	1.411	0.890	2.237	0.143				
Gender	(female vs. male)	0.876	0.588	1.306	0.517				
Venus invasion	(yes vs. No)	2.572	1.662	3.980	0.000	1.595	0.545	4.673	0.394
Perineural invasion	(yes vs. No)	1.964	0.995	3.878	0.052	1.219	0.575	2.587	0.605
T stage	(T3–4 vs. T1–2)	2.725	1.825	4.068	0.000	1.560	0.755	3.225	0.230
N stage	(N1–2 vs. N0)	2.043	1.615	2.585	0.000	1.748	1.040	2.937	0.035
M stage	(M1 vs. M0)	4.317	2.794	6.671	0.000	1.980	0.834	4.699	0.121
Tumor deposit	(yes vs. No)	1.769	0.862	3.627	0.120				
Lymphatic invasion	(yes vs. No)	2.146	1.397	3.296	0.000	0.685	0.218	2.156	0.518
NLGN1 expression	(high vs. low)	2.219	1.482	3.323	0.000	2.524	1.254	5.083	0.010

**Table 3:** Univariate analysis of the prognostic factors of DFS in CRC patients from our cohort

Factors		Univariate analysis			
		Odd ratio	95% CI		P value
Age	(per year)	1.027	0.993	1.061	0.123
Gender	(female vs. male)	0.974	0.443	2.145	0.948
T stage	(T3–4 vs. T1–2)	3.554	1.857	6.800	0.000
N stage	(N1–2 vs. N0)	1.779	1.130	2.801	0.013
M stage	(M1 vs. M0)	3.771	1.548	9.183	0.003
Pretreatment CEA level	(per ng/mL)	1.010	1.001	1.019	0.027
Pretreatment CA199 level	(per U/ml)	1.003	1.000	1.007	0.054
Histological type	(mucinous adenocarcinoma vs. adenocarcinoma)	1.679	0.629	4.480	0.301
Perineural invasion	(yes vs. No)	2.133	0.627	7.251	0.225
Venus invasion	(yes vs. No)	2.784	1.036	7.479	0.042
Tumor deposit	(yes vs. No)	11.069	3.474	35.268	0.000
Tumor location		0.807	0.454	1.435	0.466
Surgical approach	(laparoscopy vs. open)	1.799	0.773	4.184	0.173
Differentiation	(mid-high differentiation vs. low differentiation)	2.232	0.663	7.520	0.195
NLGN1 expression	(high vs. low)	2.368	1.065	5.267	0.034

### The potential functions of NLGN1 in CRC

GSEA showed that a total of 12 pathways, including “Hedgehog signaling pathway”, “Glycosaminoglycan biosynthesis heparan sulfate”, “Pyruvate metabolism”, “Terpenoid backbone biosynthesis”, “Biosynthesis of unsaturated fatty acids”, “RNA degradation”, “RNA polymerase”, “Proteasome”, “Base excision repair”, “Mismatch repair”, “Peroxisome”, and “Protein export”, were enriched and shared by all 3 datasets and are considered as the crucial signatures of NLGN1 (Table 4). Data regarding microsatellite-instability status was only collected in 94 study participants from TCGA, the analysis found that NLGN1 expression level was significantly higher in microsatellite stable (MSS) patients compared with that in microsatellite instable (MSI) patients (5.8 ± 3.6 vs. 1.8 ± 2.6, *P* = 0.001, Fig. 2D).

**Table 4:** The enriched hallmark signatures that were significantly associated with NLGN1 by Gene set enrichment analysis (GSEA)

	Gene size	Enrichment score	P value
Hedgehog signaling pathway	53	0.30	<0.001
Glycosaminoglycan biosynthesis heparan sulfate	26	−0.33	<0.001
Pyruvate metabolism	38	−0.38	<0.001
Terpenoid backbone biosynthesis	15	−0.61	<0.001
Biosynthesis of unsaturated fatty acids	19	−0.34	<0.001
RNA degradation	57	− 0.62	<0.001
RNA polymerase	28	−0.62	<0.001
Proteasome	41	−0.69	<0.001
Base excision repair	32	−0.67	<0.001
Mismatch repair	22	−0.72	<0.001
Peroxisome	77	−0.43	<0.001
Protein export	23	−0.57	<0.001

Results from analysis of GSE39582 dataset

To explore the mechanism by which NLGN1 is upregulated in CRC, we analyzed the association among mRNA expression, methylation status, copy number, and mutation status of NLGN1 in public datasets from the cbioportal database. There was no association between the methylation level and mRNA expression (Spearson test, *P* = 0.190, Fig. 6A). Mutation in NLGN1 was relatively rare with a prevalence of only 1.6% in CRC samples (Fig. 6D), and mutation was not associated with NLGN1 mRNA expression (Fig. 6B). In addition, no association between the copy number and NLGN1 mRNA expression was observed (Fig. 6C).

**Fig. 6:** The mechanism by which NLGN1 is upregulated in CRC. **A** There was no association between the methylation level and mRNA expression; **B** Mutation was not associated with NLGN1 mRNA expression. **C** No association between the copy number and NLGN1 mRNA expression was observed; **D** Mutation in NLGN1 was relatively rare with a prevalence of only 1.6% in CRC samples

## Discussion

Due to a lack of accuracy of the pathological prognostic prediction method alone in predicting prognosis of CRC [18], molecular biomarkers are used to help the stratification of higher-level phenotypic features and guide treatment strategies [19]. Currently, only KRAS and NRAS mutations are used routinely as a negative biomarker to avoid the use of anti-EGFR therapy [20]. Further study demonstrated that NRAS mutations affect metastatic CRC patients’ prognosis [21]. Over the past decade, achievements in molecular biology including the availability of large databases enable the bioinformatics analysis of the genomic landscape of CRC patients, which provided information on the unexplored moleculars deregulated in CRC [19]. The role of NLGN1 in CRC is never studied before. In the present study, basing 5 independent cohorts comprised of 1195 cases, we demonstrated that upregulated NLGN1 is associated with poor survival in CRC.

In general, NLGNs are cell-adhesion proteins that regulate synapse formation and function [22]. In humans, NLGNs family includes 5 members. NLGN1 is a major component of excitatory glutamatergic synapses complex [10]. Therefore, previous studies on NLGN1, which are preferentially expressed in human brain, focus mostly on neurodevelopmental disorders [12]. For instance, NLGN1 polymorphisms were proved to be associated with schizophrenia in Chinese Han population [12]. Mechanically, NLGNs and neurexins are located at opposite sides of synaptic membranes, and NLGNs/neurexins synaptic complex plays a role in the regulation of the schizophrenia-related protein function [23]. Several NLGN1 missense variants were found in autism patients and were demonstrated to be functionally significant in mice model [10]. To date, only two studies evaluated the role of NLGN1 in bowel diseases. Wang et al. [24] revealed that NLGN1 and glutamate may represent novel biomarkers of ganglion cells, whose expression were associated with the severity of Hirschsprung’s disease. NLGN1 and glutamate were co-expressed highest to lowest in the ganglionic, transitional and aganglionic segments. Furthermore, Xiao et al. [25] found that decreasing expressions of NLGN1 proteins induced the dysfunction of ganglion cells in distal intestinal canal, which is associated with poor prognosis of children patients with Hirschsprung’s disease after operation.

However, very few studies have been conducted to investigate NLGN1’s biological role specific to cancer. Cha et al. [26] found that NLGN1 had the highest amplification frequencies in oral squamous cell carcinoma. Davidson et al. [27] revealed that NLGN1 was overexpressed in primary uterine leiomyosarcoma. The above results suggest that NLGN1 was identified as an oncogene involves in the pathogenic process of cancers. The analysis in the present study also demonstrated that NLGN1 mRNA and protein expression was increased in CRC. Interestingly, similar to what was observed in the previous study [25], ganglion cells had positive NLGN1 protein expression in the present study. Moreover, the patients with perineural invasion had significantly higher NLGN1 expression than those without perineural invasion. As a cellular adhesion receptor, the role of NLGN1 in cancer cell migration through peripheral nerve fiber needs further investigation. The gene sets of Hedgehog (Hh) signaling pathway were enriched in the CRC tissues with high NLGN1 expression in GSEA analysis. Constitutive activation of the Hh signaling pathway contribute to tumorigenesis in various malignancies [28]. In CRC, Hh signaling is activated by both canonical signaling (via Smo) and non-canonical signaling [29]. Interestingly, GSEA of NLGN1 showed that the mismatch repair process was significantly enriched in the present study. Defects in the DNA mismatch repair proteins, result in MSI phenotype, occurring in about 15% of sporadic CRC [30]. It is known that CRCs with MSI have a significantly better survival than those with intact mismatch repair [31]. Our further analysis also detected a similar trend that NLGN1 expression was significantly lower in MSI patients, with better survival, compared with that in MSS patients. The functional enrichment analysis also revealed several metabolism pathways enriched in NLGN1. Specific metabolic activities can participate directly in the process of tumor initiation and progression [32]. However, the underlying mechanism is still needed for further investigation.

Concerning the value of NLGN1 for predicting survival, IHC analysis of patients in our centre showed that the higher NLGN1 protein was correlated with worse DFS in CRC patients. To obtain a robust conclusion, this result was externally validated in three independent datasets (GSE24551, GSE39582, and TCGA). Besides, multivariate regression confirmed NLGN1 as an independent poor prognostic factor for CRC patients in TCGA database. The substantial evidence in the present study indicated that NLGN1 could be a novel prognostic marker of poor survival in CRC patients.

Our integrative analysis revealed that neither methylation nor copy number alteration was the driver event of upregulation of NLGN1. In addition, Mutation in NLGN1 was relatively rare with a prevalence of only 1.6% in CRC samples. Thus, further research is needed to determine the mechanism by which NLGN1 is upregulated in CRC.

Our study had several limitations. First, we have tried to mine the GSE39582 and GSE24551 to perform the comparison of NLGN1 expression between normal versus colon cancer specimens. However, GSE24551 contained no normal samples for this analysis. Although GSE39582 contained 19 non-tumoral samples, no patient ID or information was provided and we failed to matched these samples with cancer tissues. On the other hand, the finding of bioinformatics analysis basing 17 pairs of samples was further confirmed at the protein level in 52 pairs of samples in our cohort. Second, the detection of NLGN1 protein was only performed in small tissue samples of 52 cases in our own cohort to investigate the effect of NLGN1 on the oncological outcome of CRC patients. However, the results were further externally validated in three independent datasets (GSE39582, GSE24551, and TCGA). Third, the detail function of NLGN1 in CRC was not evaluated. The hypothesis drawn from GSEA needs to be further confirmed by in vitro and in vivo experiments.

In conclusion, this preliminary study demonstrated that NLGN1 was up-regulated in CRC and high NLGN1 expression could be used as an independent parameter to predict the poor prognosis of CRC patients by using multiple datasets and our database. The potential function of NLGN1 in CRC was related to the Hh signaling pathway, mismatch repair process, and some material metabolism processes. Thus, NLGN1 may serve as a novel prognostic biomarker and therapeutic target for CRC.

## Data Availability

The dataset supporting the conclusions of this article is included within the article. All TCGA related data can be obtained from the TCGA Data Portal via https://tcga-data.nci.nih.gov/. All GEO related data can be obtained from the GEO Data Portal via https://www.ncbi.nlm.nih.gov/geo/.

## Abbreviations

NLGN1: Neuroligin 1
CRC: Colorectal cancer
GSEA: Gene Set Enrichment Analysis
IHC staining: Immunohistochemical staining
GEO: Gene Expression Omnibus
TCGA: The Cancer Genome Atlas
MSS: Microsatellite stable
MSI: Microsatellite instable
